The article "Deep Learning-Based Electrocardiograph in Evaluating Radiofrequency Ablation for Rapid Arrhythmia" was published in 2022. Journal: Comput Math Methods Med.

# Deep Learning-Based Electrocardiograph in Evaluating Radiofrequency Ablation for Rapid Arrhythmia

**DOI:** 10.1155/2022/6491084

**Published:** 2022-03-23

**Authors:** Guoqiang Wang, Guocai Chen, Xueqin Huang, Jianbo Hu, Xuejun Yu

**Affiliations:** Department of Cardiology, Chongqing Kanghua Zhonglian Cardiovascular Hospital, 163 Haier Road, Jiangbei District, Chongqing City 400000, China

## Abstract

This study is aimed at analyzing the important role of deep learning-based electrocardiograph (ECG) in the efficacy evaluation of radiofrequency ablation in the treatment of tachyarrhythmia. In this study, 158 patients with rapid arrhythmia treated by radiofrequency ablation were divided into effective treatment group (142 cases) and ineffective treatment group (16 cases). ECG examination was performed on all patients, and the indicators of ECG examination were quantified by the deep learning-based convolutional neural network model. The indicators of ECG examination of the effective treatment group and the ineffective treatment group were compared. The results showed that compared with the ineffective treatment group, the end-systolic volume (ESV), end-diastolic volume (EDV), end-systolic volume index (ESVI), and end-diastolic volume index (EDVI) of the effective treatment group were significantly decreased, and the left ventricular ejection fraction (LVEF) was significantly increased (*P* < 0.05). After radiofrequency ablation, the ventricular rate of patients in the effective treatment group was significantly lower than that of the ineffective treatment group at 12 h and 24 h after treatment (*P* < 0.05). In addition, compared with patients in the ineffective treatment group, the QT dispersion of the ECG in the effective treatment group was significantly higher (*P* < 0.05). The accuracy, specificity, and sensitivity of ECG in evaluating the therapeutic effect of patients with tachyarrhythmia were 86.81%, 84.29%, and 77.27%, respectively. The area under the curve was determined as 0.798 according to the receiver operating characteristic (ROC) curve of the subjects. In summary, indicators of ECG examination based on deep learning can provide auxiliary reference information for the efficacy evaluation of radiofrequency ablation in the treatment of tachyarrhythmia.

## 1. Introduction

Arrhythmia is very common in cardiovascular diseases, which can occur in the form of complications or in the form of separate existence in clinic [1]. Arrhythmias can be divided into slow onset sinus bradycardia and rapid bradycardia according to ventricular rate. Cardiac pacing point is located outside the sinus node or sinus node, and ventricular rate more than 100 times/min of arrhythmia is determined as tachyarrhythmia. In clinical practice, it is often manifested as supraventricular tachycardia, sinus tachycardia, atrial flutter, atrial fibrillation, etc. [2–4]. The clinical symptoms of this disease are chest tightness and shortness of breath. Severe patients will have hemodynamic changes; continuous development will cause the occurrence of other diseases and even the risk of sudden death [5]. A variety of factors can lead to the occurrence of rapid heart rate abnormality, including heart disease caused by heart itself and other reasons [6, 7]. Pathogenic factors can be divided into physiological and pathological two categories. Physiological factors can usually be restored by themselves without additional treatment. Physiological factors include eating habits, adequate sleep, living habits, and emotional stability. Pathological factors include cardiovascular diseases such as congenital heart disease and rheumatic heart disease; endocrine system diseases such as thyroid dysfunction and metabolic disorders; electrolyte disorders caused by serum potassium and sodium; physical and chemical factors such as freezing, surgery, and external stimulation; and the use of antiarrhythmic drugs such as digitalis and milrinone [8–10].

The article "Deep Learning-Based Electrocardiograph in Evaluating Radiofrequency Ablation for Rapid Arrhythmia" was published in 2022. Journal: Comput Math Methods Med.

With the continuous development of science and technology and medical level, a variety of methods for the treatment of tachyarrhythmia have emerged, which can be divided into drug treatment and nondrug treatment. Nondrug treatments include cardiac surgery, electrical cardioversion and defibrillation, and radiofrequency ablation [11–13]. There are four kinds of drugs for the treatment of tachyarrhythmia: class I for blocking sodium channel drugs, class II for blocking beta receptor drugs, class III for blocking myocardial potassium channel drugs, and class IV for blocking calcium channel drugs [14–16]. The continuous development and maturity of nondrug therapy have also attracted the attention of medical workers. Electro cardioversion and defibrillation are commonly used in severe tachyarrhythmias. Operating principle is to use a certain transient high voltage and strong current through the chest wall directly acting on the heart, so that most or even all of the myocardial cells instantaneous depolarization. The electrical activity of the heart stops instantly, so that the heart is redominated by the highest self-regulatory pacing point, namely, the sinus node, and the abnormal heart rhythm is transformed into the normal sinus rhythm [17, 18]. Cardiac surgery mainly improves the abnormal function of the heart to return to normal rhythm by directly cutting the tissue used for sinus velocity generation [19]. Catheter radiofrequency ablation is to send an ablation catheter into the cardiac cavity through peripheral venous blood vessels, find abnormal “excited points,” and selectively degenerate and inactivate part of the myocardial tissue that causes tachyarrhythmias to cause coagulation necrosis, thereby causing coagulation necrosis. Due to the good efficacy and safety of this treatment method, it has become a commonly used treatment method in the field of arrhythmia treatment [20–23].

The article "Deep Learning-Based Electrocardiograph in Evaluating Radiofrequency Ablation for Rapid Arrhythmia" was published in 2022. Journal: Comput Math Methods Med.

Electrocardiogram (ECG) is a technology that uses an electrocardiograph to record the changes in the electrical activity patterns of the heart during each cardiac cycle from the body surface. It is one of the most commonly used clinical examinations. It can play an important role in a variety of clinical applications, such as recording the electrical activity of the human body's normal heart, helping to diagnose arrhythmia, and judging the pacing status of artificial heart [24, 25]. By reading many extremely complex influence information from ECG examination results and establishing corresponding algorithms, further analysis and clarification can help clinicians diagnose or treat diseases more accurately and quickly and at the same time get more in-depth information about the disease [26]. Convolutional neural network is a kind of deep neural network, and its composition is a deeper grid structure. It can read the image data as visual pathological features and find the feature data that human eyes cannot read. This is very important for using ECG examination based on deep learning algorithm to analyze and evaluate the efficacy of radiofrequency ablation in the treatment of rapid arrhythmia [27–29].

In this study, 158 patients with rapid arrhythmia treated by radiofrequency ablation were divided into effective treatment group (142 cases) and ineffective treatment group (16 cases). All patients were examined by electrocardiogram. The ECG examination indexes of the effective treatment group and the ineffective treatment group were compared, and the application value of ECG examination indexes based on deep learning algorithm in evaluating the efficacy of radiofrequency ablation in the treatment of tachyarrhythmias was explored, to provide auxiliary reference information for the evaluation of the efficacy of radiofrequency ablation for the treatment of tachyarrhythmias.

## 2. Materials and Methods

### 2.1. Research Objects

In this study, 158 patients with rapid heart rate arrhythmia treated by radiofrequency ablation in hospital from January 10, 2017, to May 10, 2021, were selected. There were 90 males and 68 females, with an age range of 49-78 years old and an average age of 60.31 ± 2.7 years old. The patients were divided into effective treatment group (142 cases) and ineffective treatment group (16 cases) according to the postoperative follow-up results, whether arrhythmia control was achieved, and whether there was short-term or long-term recurrence. This study had been approved by ethics committee of hospital. The patient's family members were informed of the study and signed informed consent.

The article "Deep Learning-Based Electrocardiograph in Evaluating Radiofrequency Ablation for Rapid Arrhythmia" was published in 2022. Journal: Comput Math Methods Med.

Inclusion criteria are as follows: (1) According to the diagnostic criteria had been diagnosed with tachyarrhythmia patients, (2) the patient had been treated with radiofrequency ablation, (3) patients who had signed informed consent, and (4) patients without contraindications.

Exclusion criteria are as follows: (1) patients with other severe heart diseases, (2) patients were severely allergic, (3) patients with other serious underlying diseases, and (4) patients whose family members did not agree and did not sign informed consent.

### 2.2. Radiofrequency Ablation Therapy

The electrode catheter was inserted through skin puncture in the right internal jugular vein or left subclavian vein and right femoral vein of the patient. During the whole process, the physiological examination indexes of the patients were observed and recorded in real time, including surface electrocardiogram, his bundle, high right atrium, and coronary sinus electrogram. At the same time, electrophysiological index signals were collected to confirm the type of tachycardia in patients. After determining the target location (taking the bypass mapping as an example), the catheter was inserted into the left side of the left ventricular mitral valve to locate the ablation bypass. The right accessory pathway also inserted the catheter into the right ventricular tricuspid valve to measure the position of the ablation accessory pathway. The discharge power of the left side is set to 25-35 W, and the discharge power of the right side is set to 15-50 W. The first discharge duration is 10 s. The continuous discharge time of the target was set in the range of 30-60 to achieve the therapeutic purpose of completely blocking the bypass.

### 2.3. ECG Examination

Before the ECG examination, the examinee should be informed of the significance of the examination of the ECG that the examination is painless and harmless, to help relieve the patient's tension, relax the muscles, and lie on the examination bed in a supine state. Firstly, the ground wire and the power cord were connected well, the power switch was turned on, and the machine was preheated. The lead wires were connected according to the regulations. The examinee's bilateral wrists and the upper medial malleolus on both sides were exposed and wiped with alcohol gauze to make the skin red. Then, the conductive liquid was applied to keep the skin in good contact with the electrode. For limb lead position, the battery lead plate was connected with the ground wire in the order of the upper right limb → red line, upper left limb → yellow line, lower left limb → green line, and lower right limb → black line. Thoracic lead monitoring electrode position is as follows: V1, the fourth intercostal space on the right edge of the sternum; V2, the fourth intercostal space on the left edge of the sternum; V3, the midpoint of the connection between V2 and V4; V4, the left midclavicular line intersects with the fifth intercostal space; V5, left front axillary line V4 level; V6, left mid axillary line V4 level; V7, left posterior axillary line V4 level; and V8, left scapular line V4 level.

The article "Deep Learning-Based Electrocardiograph in Evaluating Radiofrequency Ablation for Rapid Arrhythmia" was published in 2022. Journal: Comput Math Methods Med.

### 2.4. Deep Learning Algorithm Model

The standard pattern of ECG signal contains 12 leads in total, including 8 lead orthogonal and 4 leads derived from the former. The multilead form of the ECG is similar to the two-dimensional image, and there are also differences in the data within and between the leads. According to this special lead mode, the one-dimensional convolution of the deep convolutional neural network (DCNN) can complete this type of end-to-end tasks. The network structure adopts 34-layer ResNet, changing the two-dimensional convolution in the original ResNet to one-dimensional convolution. At the same time, the size of the first layer of convolution kernel was set to 15 × 1, and the step size was designed to 2 to adapt to the input size of 2048 × 1, and the output length of the fully connected layer was set to 34 × 1, corresponding to 34 heart rate types. The specific structural model was shown in Figure 1.

ResNet, as an excellent object detection, image classification, and segmentation model, has been widely used in convolutional neural networks. ResNet model has residual structure, which makes it easier to optimize. In the propagation process of neural networks, the propagation gradient gradually disappears due to the emergence of reverse propagation. The existence of residual structure solves this problem. The gradient information of residual structure is easier to spread in the process of reverse propagation. Therefore, the network with residual module will also get higher recognition accuracy. At the same time, ResNet residual network model adopted a large number of more standardized methods for enzyme training. The specific residual unit was shown in Figure 2.

ResNet improves the number of network layers by residual structure and simplifies the learning object. The training speed and parameter accuracy are improved. The initial value *x*_*i*_ is input. The weight is set to *a*. The bias is represented by *c*, and *y*_*i*_ is a branch. The calculation functions are as follows:

(1) $$\begin{array}{c} F\left(x_{i}\right)=ax_{i}+c, \end{array}$$

(2) $$\begin{array}{c} y_{i}=M\left(F\right)+v\left(x_{i}\right), \end{array}$$

(3) $$\begin{array}{c} x_{i+1}=M\left(y_{i}\right). \end{array}$$

The activation function can avoid the gradient dispersion problem and reduce the gradient attenuation. Its equation is expressed as follows:

(4) $$\begin{array}{c} M\left(b\right)=\max\left(0,b\right). \end{array}$$

When *b* > 0, *M* (*b*) = *b*, the derivative is 1. When *b* < 0, *M* (*b*) = 0, the derivative is 0. When *b* = 0, *M* (*b*) = 0, the derivative is 0.

The article "Deep Learning-Based Electrocardiograph in Evaluating Radiofrequency Ablation for Rapid Arrhythmia" was published in 2022. Journal: Comput Math Methods Med.

Cross entropy is a loss function, where *o* and *p* are two normal probability distributions. The cross entropy of *o* is represented by *p*. Its equation is expressed as follows:

(5) $$\begin{array}{c} M\left(o,p\right)=-\sum o\left(a\right)\log p\left(a\right). \end{array}$$

As shown in equation (6) and equation (7), the cross entropy must satisfy the probability distribution function.

(6) $$\begin{array}{c} \forall ao\left(X-a\right)\in \left[0,1\right], \end{array}$$

(7) $$\begin{array}{c} \sum o\left(X-a\right)=1. \end{array}$$

### 2.5. Evaluation Indicators

The basic data of the two groups of patients were compared and analyzed, including age, heart rate, body mass index, hypertension, diabetes, smoking, drinking, and vascular history. The overall cardiac function parameters of the two groups were obtained, including left ventricular ejection fraction (LVEF), right ventricular ejection fraction (RVEF), end-systolic volume (ESV), end-diastolic volume (EDV), end-systolic volume index (ESVI), and end-diastolic volume index (EDVI). The differences of parameters between the two groups were compared and analyzed. The changes of heart rate and ECG QT dispersion after radiofrequency ablation were compared between the two groups. This study took the grouping basis of effective treatment and ineffective treatment as the reference standard. Three common indicators were used to evaluate the ability of indicators of ECG examination to assess the therapeutic effect of patients with tachyarrhythmia. They were accuracy, specificity, and sensitivity. The calculation methods are shown in equation (8), equation (9), and equation (10), respectively.

(8) $$\begin{array}{c} \text{Accuracy}=\frac{A+B}{A+C+B+D}, \end{array}$$

(9) $$\begin{array}{c} \text{Specificity}=\frac{B}{C+B}, \end{array}$$

(10) $$\begin{array}{c} \text{Sensitivity}=\frac{A}{D+A}. \end{array}$$

Among them, *A* was true positive, indicating that the diagnosis result was positive, and it was actually positive. *B* referred to true negative, indicating that the diagnosis result was negative and was actually negative. *C* was false positive, meaning that the diagnosis is positive and actually negative. *D* was false negative, indicating that the actual result was positive, and the diagnosis result was negative.

The article "Deep Learning-Based Electrocardiograph in Evaluating Radiofrequency Ablation for Rapid Arrhythmia" was published in 2022. Journal: Comput Math Methods Med.

Receiver operating characteristic (ROC) curves were used to represent the ability of indicators of ECG examination to assess therapeutic efficacy in patients with rapid arrhythmia. Area under curve (AUC) was determined according to ROC.

### 2.6. Statistical Methods

The SPSS software was used for statistical analysis of data. The data in line with normal distribution were expressed as mean ± standard deviation (mean ± s). *t*-test was used to represent the measurement data, chi-square (*χ*2) test was used to represent the count data, and *P* < 0.05 indicated that there was statistical difference.

## 3. Results

### 3.1. ECG Examination Results of Patients with Tachyarrhythmia

Figure 3 shows the ECG results of a patient with atrial arrhythmia, male, 62 years old. The results showed that the patient had multifocal atrial tachycardia, and the continuous action potentials generated by multiple abnormal areas in the atrium were all conducted to the ventricles. As a result of this, the ectopic P wave originating outside the sinus node showed irregular changes.

### 3.2. Comparison of Basic Data between the Two Groups of Patients

The basic data of the two groups were compared, and it was found that there was no significant difference in age, body mass index, hypertension, diabetes, smoking, drinking, and vascular history between the two groups (*P* > 0.05). The average heart rate of patients in the effective treatment group was significantly lower than that in the ineffective treatment group (*P* < 0.05). The specific results are shown in Figure 4.

### 3.3. Comparison of Cardiac Function Parameters

The cardiac function parameters of the two groups before and after treatment were obtained. Comparative analysis showed that EDV, EDVI, ESV, and ESVI in the effective treatment group were significantly decreased after treatment, and LVEF was significantly increased (*P* < 0.05). There was no significant difference in RVEF, RVEDV, and RVESV parameters before and after treatment (*P* > 0.05). In addition, compared with the ineffective treatment group, the parameters of EDV, EDVI, ESV, and ESVI in the effective treatment group were significantly decreased, while LVEF was significantly increased (*P* < 0.05). There were no significant differences in RVEF, RVEDV, and RVESV (*P* > 0.05). The results are shown in Figure 5.

The article "Deep Learning-Based Electrocardiograph in Evaluating Radiofrequency Ablation for Rapid Arrhythmia" was published in 2022. Journal: Comput Math Methods Med.

### 3.4. Comparison of Heart Rate and QT Dispersion Degree of Electrocardiogram between the Two Groups

The ventricular rate and QT dispersion of the ECG at 12 h and 24 h after treatment were compared between the two groups of patients. The results showed that the ventricular rate of the effective treatment group was significantly lower than that of the ineffective treatment group at 12 h and 24 h after treatment (*P* < 0.05). In addition, compared with patients in the ineffective treatment group, the QT dispersion of the ECG in the effective treatment group was significantly higher (*P* < 0.05). The results are shown in Figure 6.

### 3.5. Evaluation Efficiency of Indicators of ECG Examination

By calculating accuracy, specificity, and sensitivity, it was found that the accuracy, specificity, and sensitivity of indicators of ECG examination in evaluating the therapeutic effect of tachyarrhythmia patients were 86.81%, 84.29%, and 77.27%, respectively. The results are shown in Figure 7.

The specificity and sensitivity of radiofrequency ablation for tachyarrhythmia patients were evaluated based on indicators of ECG examination, and ROC curves were drawn, as shown in Figure 8. Meanwhile, AUC was determined to be 0.798 according to ROC.

## 4. Discussion

At present, tachyarrhythmia is a common cardiovascular disease in various populations and has become one of the heart diseases that threaten human health. Patients with rapid arrhythmia often show heart failure, hemodynamic disorders, and even shock. It threatens human life and health at all times, and the disease has become the main factor causing human death [30]. In the United States, the number of sudden cardiac death caused by tachyarrhythmias is about 300,000 people/year, according to research reports [31]. Radiofrequency ablation has gradually become a common method for the treatment of tachyarrhythmia since its first application. It has two main advantages: high success rate and small trauma. Radiofrequency ablation at the same time will not be affected by age or other basic organic heart disease images. Radiofrequency ablation has become the preferred method to cure tachyarrhythmia. The efficacy evaluation of radiofrequency ablation in the treatment of tachyarrhythmia is particularly important [32, 33]. As a kind of deep neural network, convolutional neural network can convert image data into visual pathological features and obtain information that cannot be directly captured by the human eyes. At the same time, the image information can be transformed into quantitative data to achieve the purpose of accurately reading image features. The development status of diseases can be quantitatively evaluated [34].

The article "Deep Learning-Based Electrocardiograph in Evaluating Radiofrequency Ablation for Rapid Arrhythmia" was published in 2022. Journal: Comput Math Methods Med.

This study is aimed at analyzing the important role of ECG examination based on deep learning in the efficacy evaluation of radiofrequency ablation in the treatment of tachyarrhythmia and providing effective theoretical reference for the efficacy of radiofrequency ablation. In this study, 158 patients with rapid arrhythmia treated by radiofrequency ablation were divided into effective treatment group (142 cases) and ineffective treatment group (16 cases). There were no significant differences in age, body mass index, hypertension, diabetes, smoking, drinking, and vascular history between the two groups (*P* > 0.05). The average heart rate of the effective treatment group was significantly lower than that of the ineffective treatment group (*P* < 0.05). ECG examination was performed on both groups of patients, and the indicators of ECG examination were quantified by convolution neural network model of deep learning algorithm. The indicators of ECG examination of patients in the effective treatment group and the ineffective treatment group were compared to evaluate the application value of ECG based on deep learning algorithm in evaluating the therapeutic effect of radiofrequency ablation on tachyarrhythmia. It was found that EDV, EDVI, ESV, and ESVI in the effective treatment group were significantly decreased after treatment, while LVEF was significantly increased (*P* < 0.05). There were no significant differences in RVEF, RVEDV, and RVESV parameters before and after treatment (*P* > 0.05), which may be due to the fact that the sample size collected is too small and the experimental results are biased. In addition, compared with the ineffective treatment group, the parameters of EDV, EDVI, ESV, and ESVI in the effective treatment group were significantly decreased, while LVEF was significantly increased (*P* < 0.05). There were no significant differences in RVEF, RVEDV, and RVESV (*P* > 0.05). These results are consistent with the conclusion drawn by Zhu et al. [35] that cardiac function parameters such as EDV, EDVI, ESV, ESVI, and LVEF are related to the efficacy of RFA. In addition, the ventricular rate and QT dispersion of the ECG at 12 h and 24 h after treatment were compared between the two groups. The results showed that the ventricular rates of patients in the effective treatment group were significantly lower than those in the ineffective treatment group at 12 h and 24 h after treatment (*P* < 0.05); in addition, compared with patients in the ineffective treatment group, the QT dispersion of the ECG in the effective treatment group was significantly higher (*P* < 0.05). By calculating accuracy, specificity, and sensitivity, it was found that the accuracy, specificity, and sensitivity of indicators of ECG examination in evaluating the therapeutic effect of tachyarrhythmia patients were 86.81%, 84.29%, and 77.27%, respectively. ECG shows high accuracy, specificity, and sensitivity in evaluating the efficacy of patients with tachyarrhythmias. The AUC-ROC curve is a performance measure for classification problems under various threshold settings, ROC is a probability curve, AUC represents the degree or measure of separability, and the higher the AUC, the better it can distinguish disease from disease-free. In this work, the AUC was determined to be 0.798 according to the ROC, indicating that the ECG examination index had a good evaluation effect on the efficacy of RFA in patients with tachyarrhythmias. These results revealed that indicators of ECG examination can provide a reference for evaluating the efficacy of radiofrequency ablation for tachyarrhythmia. Aryana et al. [36] applied ECG examination to observe the efficacy of amiodarone in the treatment of tachyarrhythmias and found that ECG examination information can provide a quantitative reference for the effect of drug treatment and help evaluate the condition of patients after treatment. Such results are similar to those of this work. In conclusion, ECG examination based on deep learning can provide auxiliary information for the efficacy evaluation of radiofrequency ablation for tachyarrhythmia and has great application value.

The article "Deep Learning-Based Electrocardiograph in Evaluating Radiofrequency Ablation for Rapid Arrhythmia" was published in 2022. Journal: Comput Math Methods Med.

## 5. Conclusions

In this work, 158 patients with tachyarrhythmias treated by RFA were selected for ECG examination, and the ECG examination indexes of the effective treatment group and the ineffective treatment group were compared. The results showed that multiple cardiac function parameters were related to the efficacy of RFA. In addition, the ECG examination indexes showed high accuracy, specificity, and sensitivity in evaluating the efficacy of patients with tachyarrhythmias. The shortcomings of this work were that the sample size of the research object was small, the source was single, and the randomness and wide applicability were not high. In follow-up studies, multisite, multitype, large-sample analyses and studies would be considered. This work could provide a more practical and effective reference value for the application of ECG examination indicators in evaluating the efficacy of RFA.

## Figures and Tables

**Figure 1:** Schematic diagram of the improved ResNet model structure.

**Figure 2:** The specific residual unit.

**Figure 3:** ECG examination results of patients with tachyarrhythmia.

**Figure 4:** Comparison results of basic data of two groups of patients: (a) the comparison results of age, heart rate, and body mass index between the two groups; (b) the result of comparing the proportion of patients with hypertension, diabetes, smoking, drinking, and vascular diseases between the two groups. ^∗^ expresses significant differences, *P* < 0.05.

The article "Deep Learning-Based Electrocardiograph in Evaluating Radiofrequency Ablation for Rapid Arrhythmia" was published in 2022. Journal: Comput Math Methods Med.

**Figure 5:** Comparison of cardiac function parameters between the two groups before and after treatment: (a, b) the comparison results of EDV, EDVI, ESV, ESVI, LVEF, RVEF, RVEDV, and RVESV cardiac function indexes between the two groups before treatment; (c, d) the results of EDV, EDVI, ESV, ESVI, LVEF, RVEF, RVEDV, and RVESV cardiac function indexes before and after treatment in effective treatment group. ^∗^ represents significant difference, *P* < 0.05.

**Figure 6:** Comparison results of ventricular rate (a) and electrocardiogram QT dispersion (b) of patients in the two groups. In (b), the abscissa Pre represents pretreatment, and Post represents posttreatment. ^∗^ represents significant difference, *P* < 0.05.

**Figure 7:** Evaluation of indicators of ECG examination on the efficacy of radiofrequency ablation.

**Figure 8:** ROC curve results of indicators of ECG examination based on deep learning algorithm.

## Data Availability

The data used to support the findings of this study are available from the corresponding author upon request.
